# Gene Differential Expression and Interaction Networks Illustrate the Biomarkers and Molecular Biological Mechanisms of Unsaponifiable Matter in Kanglaite Injection for Pancreatic Ductal Adenocarcinoma

This article has been retracted.

**DOI:** 10.1155/2022/6229462

**Published:** 2022-06-06

**Authors:** Bowen Xu, Wenchao Dan, Xiaoxiao Zhang, Heping Wang, Luchang Cao, Shixin Li, Jie Li

**Affiliations:** ^1^Department of Oncology, Guang'anmen Hospital, China Academy of Chinese Medical Sciences, Beijing 100053, China; ^2^Beijing University of Chinese Medicine, Beijing 100029, China; ^3^Department of Dermatological, Beijing Hospital of Traditional Chinese Medicine, Capital Medical University, Beijing 100010, China

## Abstract

**Background:**

Kanglaite injection (KLTi) has shown good clinical efficacy in the treatment of pancreatic ductal adenocarcinoma (PDAC). While previous studies have demonstrated the antitumor effects of the oil compounds in KLTi, it is unclear whether the unsaponifiable matter (USM) also has antitumor effects. This study used network pharmacology, molecular docking, and database verification methods to investigate the molecular biological mechanisms of USM.

**Methods:**

Compounds of USM were obtained from GC-MS, and targets from DrugBank. Next, the GEO database was searched for differentially expressed genes in cancerous tissues and healthy tissues of PDAC to identify targets. Subsequently, the protein-protein interaction of USM and PDAC targets was constructed by BisoGenet to extract candidate genes. The candidate genes were enriched using GO and KEGG by Metascape, and the gene-pathway network was constructed to screen the key genes. Molecular docking and molecular dynamic simulations of core compound targets were finally performed and to explore the diagnostic, survival, and prognosis value of targets.

**Results:**

A total of 10 active compounds and 36 drug targets were screened for USM, 919 genes associated with PDAC, and 139 USM candidate genes against PDAC were excavated. The enrichment predicted USM by acting on *RELA*, *NFKB1*, *IKBKG*, *JUN*, *MAPK1*, *TP53*, and *AKT1*. Molecular docking and dynamic simulations confirmed the screened core targets had good affinity and stability with the corresponding compounds. In diagnostic ROC validation, the above targets have certain accuracy for diagnosing PDAC, and the combined diagnosis is more advantageous. As the most diagnostic value of *RELA*, it is equally significant in predicting disease-specific survival and progression-free interval.

**Conclusions:**

USM in KLTi plays an anti-PDAC role by intervening in the cell cycle, inducing apoptosis, and downregulating the NF-*κ*B, MAPK, and PI3K-Akt pathways. It might participate in the pancreatic cancer pathway, and core target groups have diagnostic, survival, and prognosis value biomarker significance.

## 1. Introduction

Pancreatic ductal adenocarcinoma (PDAC) is a malignant tumor of the digestive tract and accounts for about 90% of all pancreatic cancers (PC). The five-year relative survival rate for PDAC is only 9% [1]. At present, the incidence and case fatality rates of PDAC continue to rise, and it is expected to become the second leading cause of cancer-related deaths in 2030 [2]. About 90% of the patients with PDAC are diagnosed at an advanced stage, and only 20% of the patients receive surgical treatment. Moreover, the surgical resection rate of PDAC is low, and the five-year survival rate of patients with complete resection is 27% [3]. PDAC is highly metastatic and develops drug resistance easily. Due to the low efficacy and high toxicity associated with chemoradiotherapy [4], the conventional treatment modalities for PDAC have run into a bottleneck. Therefore, it is of great clinical significance and practical value to seek a safe and efficacious adjuvant therapy for PDAC.

Numerous studies have indicated that traditional Chinese medicine (TCM) has been shown to play an active role in the adjuvant treatment of PDAC by reducing the toxic effects and side effects associated with modern medical treatment [5], improving the quality of life, and prolonging the survival of patients [6]. Kanglaite injection (KLTi) is a neutral oil extracted and isolated from the seeds of the Chinese herbal medicine, *Coix lacryma-jobi* L.. It has been widely used in China as adjuvant therapy for the treatment of various advanced malignant tumors and has shown anticachexia and analgesic effects.

In mechanism research [7], KLTi has shown antitumor activity in mouse models of PDAC by inhibiting proliferation and metastasis and inducing apoptosis and necrosis. A phase II clinical trial showed that the combination of KLTi and gemcitabine in PDAC presented a difference in progression-free survival (114 days versus 57.7 days, *P* = 0.0080) and objective response rate [8], but it was fully sponsored by KLT company and may lead to the existence of conflicts of interest. To further confirm the ability of KLTi in improving the efficacy of PDAC, a meta-analysis showed that the combination of KLTi and chemoradiotherapy is more effective than chemoradiotherapy alone in the treatment of advanced PDAC. The combination treatment not only improved the 1-year overall survival rate, overall response, and disease control rate but also enhanced the quality of life, relieving pain, and alleviated adverse reactions [9]. In addition, a network meta-analysis was performed to assess the effectiveness and safety of Chinese herbal injections combined with chemotherapy for the treatment of PC. The results demonstrated that Kanglaite injection combined with chemotherapy yielded a significantly higher probability of improving performance status [10].

Further exploration of KLTi is expected to provide benefit in improving the comprehensive treatment of PDAC. A total of 12 triglycerides were identified as the main compounds in KLTi by high-performance liquid chromatography-atmospheric pressure chemical ionization-mass spectrometry (HPLC-MS) [11]. While the oily compounds in KLTi have been studied well, there are few studies on the unsaponifiable matter (USM) in KLTi. Whether these USM also have antitumor effects need further investigation.

Network pharmacology is based on various types of biological information databases. Through the network analysis of drugs, genes, compounds, and diseases and thoroughly examining the key nodes in the network [12], it is possible to systematically explain the material basis and mechanism of action of TCM [13]. Network pharmacology also emphasizes the study of multitarget pathways, which is consistent with the overall concept of TCM. Hence, it is currently used to investigate the mechanism of action and new drug development of TCM and its compound prescriptions, especially in cancer treatment [14]. Therefore, in this study, the network pharmacology and molecular docking method were used to elucidate the specific molecular biological mechanisms of USM in KLTi intervention in PDAC. And The Cancer Genome Atlas (TCGA) database was used to analyze the diagnostic effect of core targets on PDAC and the predictive effect on long-term survival.

## 2. Materials and Methods

### 2.1. Screening of Active Compounds and Targets in Unsaponifiable Matter

The USM in KLTi was separated, and their main compounds were identified by gas chromatography-mass spectrometric (GC-MS) [15]. Next, we identified the total chemical composition of *Coix lacryma-jobi* L. from the Traditional Chinese Medicine Database and Analysis Platform (TCMSP) [16] and HERB. According to the ADME (absorption, distribution, metabolism, and excretion) screening principle, there are two core indicators, oral bioavailability (OB) and drug-likeness (DL), used for screening compounds. Since KLTi is administered intravenously, it did not require screening of OB, which is specific to orally administered drugs. The screening condition for DL was set as ≥0.18. Compounds related to *Coix lacryma-jobi* L. that demonstrated antitumor activity, as confirmed from previous studies, were collected to supplement and improve the results and obtain candidate compounds.

Candidate compounds were then matched to drug targets in the DrugBank database [17] and corrected to standard gene names, using the Uniprot database [18]. Cytoscape 3.7.2 was employed to construct a compound-target network of KLTi for the selected compounds and targets [19]. The network was analyzed to analyze the relationship between the important compounds and targets in KLTi, with the help of Cytoscape's built-in network analyzer tool, focusing on the degree of connectivity. The more connected the degree, the higher importance involved in biological functions. The workflow of the network pharmacology analysis performed in this study is depicted in Figure 1.

### 2.2. Identification of PDAC-Related Targets

The differential expressed genes in cancerous tissues and healthy tissues of PDAC patients were obtained from the Gene Expression Omnibus (GEO) [20] series (GSE15471, samples: GSM388115-GSM388153 and GSM388076-GSM388114). Disease targets of PDAC were screened under the conditions of adjusted *P* value < 0.05 and |logFC| > 1, and the gene markers with significant differentially expressed genes corresponded to gene names.

### 2.3. Construction of Protein-Protein Interaction

Based on the built-in function of BisoGenet in Cytoscape 3.7.2, the protein-protein interaction (PPI) network between KLTi USM and PDAC was constructed and visualized. The intersection network of two PPI networks was extracted by the merge function, and the attribute values of each node in the intersection network were analyzed using CytoNCA [21]. The median *k*1 of the connectivity degree was calculated, and all nodes with a connectivity degree greater than 2 times *k*1 were selected and termed as “Hit hubs.” The properties of each node of the Hit hubs network were calculated to obtain three medians *k*2, *l*2, and *m*2 for connectivity degree centrality (DC), closeness centrality (CC), and betweenness centrality (BC), respectively. All nodes whose node properties were simultaneously greater than *k*2, *l*2, and *m*2 were screened as candidate targets.

### 2.4. Pathway Enrichment Analysis

The Metascape platform integrates several reliable databases such as gene ontology (GO) and Kyoto Encyclopedia of Genes and Genomes (KEGG) for pathway enrichment analysis of gene targets and is updated monthly to ensure data accuracy [22]. GO utilizes three parameters; namely, molecular function, biological process, and cellular component to interpret the antitumor biological process of candidate genes. KEGG analysis examines the main antitumor signaling pathways involved in candidate genes. The 20 GO and KEGG processes, with significant differences, were screened, and the results were visualized and analyzed with R software. Based on the relevant targets mapped by KEGG results, a gene-pathway network was constructed to further screen key target genes for KLTi treatment of PDAC.

### 2.5. Molecular Docking

#### 2.5.1. Preparation of Protein

The crystal structure of the protein was downloaded from RCSB PDB (Protein Data Bank) [23]. GUI-based “Auto-Dock Tools” was used to prepare and execute the docking studies. Kollman atom charges, solvation parameters, and polar hydrogens were added to the protein and proceeded for docking studies. As the ligands used are not peptides, Gasteiger charges were assigned only to the protein, and the nonpolar hydrogens were merged. Based on the reference ligand, literature, and predicted active regions, a grid box was assigned around the active sites using the AutoGrid application.

#### 2.5.2. Preparation of Ligand

The 3D structures of the main compounds were retrieved from the PubChem database. Minimize the energy of the downloaded compound through Chem3D and convert it into mol2 format. Import the small molecular compound into Auto-Dock Tools software, add atomic charge, and assign an atomic type [21]. All flexible keys are rotatable by default. Finally, the best conformation was retained in pdbqt format for utilization in further docking studies.

### 2.6. Molecular Dynamic Simulation

MD simulations of protein complexes with compounds were performed using Desmond (version 2020). Here, the molecular force field for MD simulations was chosen as OPLS3e, and the system was solvated using the TIP3 water model. Neutralize system charge by adding ions. The energy minimization of the whole system is achieved using the OPLS3e force field (all-atom type force field). The geometry of water molecules, bond lengths, and bond angles of heavy atoms are all constrained by the SHAKE algorithm. The continuous system is simulated by applying periodic boundary conditions, and long-range electrostatics are maintained by the particle mesh Ewald method. The system was equilibrated using an NPT ensemble with a temperature of 300 k and a pressure of 1.0 bar. The Berendsen coupling algorithm was used for the coupling of temperature-pressure parameters. At the time of late preparation of the system, 200 ns runs were performed at a time step of 1.2 fs, and trajectory recording was performed every 100 ps for a total of 20,00 frames. The RMSD (root mean square deviation) of the main chain atoms was calculated and graphically analyzed to understand the nature of protein-ligand interactions.

### 2.7. Diagnostic, Survival, and Prognosis Value Analysis of Key Targets

ROC curves were made using key target genes in combination with the data set to determine the diagnostic value for PDAC. Then, combined with the data of the GEO and TCGA database and RNAseq data from the PAAD (pancreatic cancer) project. Log-rank test with Cox regression was used. Suppose *P* < 0.05, the difference in the survival time distribution of the groups was statistically significant. Thus, the survival and prognosis analyses of the core targets obtained by the screening are carried out.

## 3. Results

### 3.1. Active Compounds of Unsaponifiable Matter

According to the GC-MS results of USM in KLTi, 10 compounds were included and queried for their DL values. A total of 38 compounds were identified in TCMSP and HERB, based on the chemical composition of *Coix lacryma-jobi* L.. Candidate compounds with DL ≥ 0.18 (18 active compounds) were included in the study. Two compounds, olein and mboa, which had demonstrated antitumor activity in previous studies [24], were excluded since their DL < 0.18. A total of 36 drug targets were matched in the DrugBank database. Of these, 10 active compounds were mapped to the corresponding targets, while 8 compounds did not match any target (Figure 2(a)). Pharmacotoxicology is commonly used to evaluate the safety profile of compounds. The protox II webserver was used to predict toxicological parameters such as hepatotoxicity, carcinogenicity, immunotoxicity, mutagenicity, cytotoxicity, and acute oral toxicity (LD50, mg/kg). None of the compounds in USM showed hepatotoxicity and mutagenicity, and 2-monoolein also presented inactive in toxicological parameters. Meanwhile, stigmasterol, sitosterol alpha1, isoarborinol, CLR, omaine, ergosterol, sitosterol, campesterol, and 2-monoolein have the risk of immunotoxicity. Mandenol has the risk of carcinogenicity, while omaine has cytotoxicity. Moreover, ergosterol and omaine showed the lowest LD50 values (10 mg/kg, 26 mg/kg) (Figure 2(b)). The chemical structure and DL of 10 compounds from USM are shown in Figure 2(c). All the compounds displayed favorable DL parameters (shown in red font). These results indicate that these 10 compounds showed good pharmacological parameters and molecular properties, which could be used as active compounds for follow-up analysis.

### 3.2. Unsaponifiable Matter and PDAC-Related Targets

A compound-target network was constructed for USM (Figure 3(a)), the nodes represented compounds or targets, and the edges represented the relationship of interactions. This network contained 46 nodes (10 compounds and 36 targets) and 64 edges. The top four key active compounds in USM were stigmasterol, mandenol, sitosterol alpha1, and isoarborinol, and their respective degrees were 26, 20, 5, and 5.

A total of 919 PDAC-related targets were identified from the GEO database. Among these, 709 were upregulated genes, and 210 were downregulated genes. A volcano plot was created to show the distribution of differentially expressed genes (Figure 3(b)), and a heat map of expression for these differential genes is shown in Figure 3(c).

### 3.3. Candidate Genes for Unsaponifiable Matter Treatment of PDAC

The PPI networks found that the drug targets of USM had a relationship with 1,966 targets, and 45,343 interrelationships existed among these targets. The PPI network of PDAC was found to contain 7,983 targets (nodes) and 17,6870 interrelationships (edges). The above two PPI networks were merged to reveal the specific targets of USM intervention in PDAC. This network, consisting of 1,558 nodes and 40,405 edges, is presented in Figure 4(a). According to data statistics, the median degree of all nodes was 37, which was filtered with DC > 68 to obtain Figure 4(b). The final candidate genes were screened and 139 targets, with DC > 103, BC > 156.4916701, and CC > 0.547414, were identified, as shown in Figure 4(c).

Since the roles of proteins in PPI networks are reciprocal, they are usually classified as undirected graphs. The presence of regions with high partial density in complex networks of PPI is referred to as a module. The network inside the module is the potential subnetwork of the PPI network, which has a higher density of subnetwork connections and fewer regional partial connections. Thus, the module can be considered a biologically meaningful set, which has two components. First is the protein complex, consisting of multiple proteins to form a complex, which subsequently plays a biological role. The other is the functional module, comprising proteins located in the same pathway but with closer interactions. Therefore, to analyze the mechanism of USM in the treatment of PDAC more precisely, it was necessary to further identify its module after obtaining the core PPI network. The module was obtained by analyzing the interaction relationship through the molecular complex detection algorithm, as shown in Figure 5. Based on the Log10*P* value, the biological processes of the top three scores in the module were retained and functionally described, as shown in Table 1.

### 3.4. GO and KEGG Pathway Enrichment

Metascape platform was used to perform GO and KEGG pathway analysis of the 139 identified candidate genes. The GO results of candidate genes showed that a total of 1,762 GO terms were significantly enriched, including 1,520 in biological processes, 133 in cellular compositions, and 109 in molecular functions. KEGG results for candidate genes revealed 119 significantly enriched pathways. According to the log10 (false discovery ratio (FDR)) value ranking, the 20 genes or pathways were selected (Figure 6).

### 3.5. Gene-Pathway Network

The gene-pathway network was constructed based on the significant difference in KEGG pathways and genes that regulated these pathways. It included 20 pathways, 57 genes, and 253 relationships (Figure 7). From the network, it was observed that *RELA* and *NFKB1* had the largest degree (19). The other genes with large degrees were *IKBKG*, *JUN*, *MAPK1*, *AKT1*, and *TP53* (17, 16, 15, 12, and 10, respectively).

### 3.6. Molecular Docking and Molecular Dynamic Simulation Analysis of Compound-Targets

Docking calculations were performed between *JUN*, *MAPK1*, *TP53*, *RELA* (PDB ID: 5AEP, 2OJG, 5BUA, and 1VJ7) and stigmasterol, isoarborinol using AutoDock4.2 to compute the free energy of binding on protein model. Essential hydrogen atoms, Kollman united atom type charges, and solvation parameters were added with the aid of AutoDock tools. Affinity (grid) maps of $60\times 60\times 60\;\overset{{}^{\circ}}{A}$ grid points and 0.375 Å spacing were generated using the AutoGrid program. AutoDock parameter set and distance-dependent dielectric functions were used in the calculation of the Van der Waals and the electrostatic terms, respectively. Docking simulations were performed using the Lamarckian genetic algorithm (LGA) and the Solis and Wets local search method. The initial position, orientation, and torsions of the ligand molecules were set randomly, and all rotatable torsions were released during docking. Each docking experiment was derived from 100 different runs that were set to terminate after a maximum of 250000 energy evaluations. The population size was set to 150. During the search, a translational step of 0.2 Å and quaternion and torsion steps of 5 was applied. Then, we used an RMSD plot during molecular dynamic simulations of core compound targets, as shown in Table 2 and Figures 8 and 9.

### 3.7. Diagnostic ROC Analysis of Key Targets

In predicting the outcomes of cancerous tissues and healthy tissues, the predictive ability of *RELA* and *TP53* had certain accuracy (AUC = 0.811, CI = 0.713–0.910; AUC = 0.723, CI = 0.607–0.839), the remaining 5 were low accuracy. Unlike before, the predictive ability of the 7-genes combination also had certain accuracy, and their values were higher than those of single-gene prediction (AUC = 0.892, CI = 0.820–0.964), which had certain clinical predictive value (Figure 10).

### 3.8. Survival and Prognosis Analysis of Key Target

In predicting the outcomes of survival and prognosis in PDAC, the predictive ability of *RELA* had high accuracy (AUC = 0.926, CI = 0.897 – 0.955). In disease-specific survival and progress free interval, low expression of *RELA* has a higher predictive value than high expression of patient viability (*P* = 0.027, HR: 1.98 (1.08–3.62); *P* = 0.003, HR: 2.25 (1.32–3.81)), especially in progress free interval. However, there was no significant difference in overall survival between high and low *RELA* expression (*P* = 0.087, HR: 1.55 (0.94–2.55)), but there was a trend towards larger spacing (Figure 11).

## 4. Discussion

In this research, we found that USM achieved a synergistic effect through multiple compounds, targets, and pathways. Molecular docking and molecular dynamic simulations showed good affinity and stability of core compound targets. The diagnostic ROC results confirmed that *RELA* and *TP53* had some accuracy in the diagnostic prediction of PDAC, and the diagnosis of combined key gene groups had more advantages, providing a basis for screening new biomarkers. We also found that *RELA* expression differed most in cancerous tissues and healthy tissues. It has also been similarly found in survival prognosis analysis that *RELA* is significant in predicting disease-specific survival and progress-free interval and can be considered as the prognostic predictors of PDAC in the future.

### 4.1. Potential Active Compounds with Antitumor Effects

The top four compounds obtained from the compound-target network of USM were stigmasterol, mandenol, sitosterol *α*1, and isoarborinol. Stigmasterol and sitosterol *α*1 belong to the class of phytosterols as anticancer dietary components [25]. Stigmasterol inhibited lipopolysaccharide- (LPS-) induced innate immune responses in murine models [26], significantly reduced the transcription level of TNF-*α*, destroyed tumor angiogenesis, and reduced the chance of metastasis [27]. Although there is insufficient data on sitosterol *α*1, related subclasses such as *β*-sitosterol and *γ*-sitosterol have demonstrated obvious anticancer effects [28, 29], and the level changes of *β*-sitosterol can significantly distinguish PC patients from healthy controls[30]. Modern pharmacological studies have confirmed that isoarborinol can be used to improve anxiety, depression, and pain. Moreover, it has an auxiliary effect on the clinical symptoms, which are prone to occur during the development of cancer treatment [31]. In the case of mandenol, there is currently no relevant clinical or experimental research data available, which can be used as a potential antitumor compound for further study.

### 4.2. Potential Gene Targets with Molecular Docking, Survival, and Prognosis Analysis

From the gene-pathway network, it was found that *RELA*, *NFKB1*, *IKBKG*, *JUN*, *MAPK1*, *TP53*, and *AKT1* were the genes with the highest interactions and were identified as potential gene targets for USM intervention in PDAC. The screened core targets were found to have good affinity and stability to the corresponding compounds, suggesting that the screening results have some reliability. Among these genes, *RELA*, *NFKB1*, and *IKBKG* are all components of the NF-*κ*B signaling pathway. The NF-*κ*B signaling pathway is one of the major signaling pathways linking cancer to inflammation. This classical pathway is activated when the cells are exposed to inflammatory cytokines, such as TNF*α* and IL-1, or in response to inflammatory signals, such as LPS [32]. In addition to inhibiting tumor cell proliferation and metastasis, NF-*κ*B also interferes with inflammation [33]. Specifically, for PDAC with pancreatitis, intervention with the NF-*κ*B signaling pathway can simultaneously result in tumor and tumor-related inflammation [34]. NF-*κ*B also helps TNF-*α* to induce epithelial-mesenchymal transition (EMT) and complete angiogenesis and metastasis. Thus, KLTi could curb tumor progression by inhibiting the NF-*κ*B signaling pathway.

*RELA* can promote PDAC progression by activating proliferation or migration-related gene expression. The binding of miR-302a-3p to *RELA* inhibited *RELA* expression as well as PDAC cell proliferation and migration [35]. This suggests that the overexpression of *RELA* promotes proliferation and metastasis of PDAC cells. Tumor suppression, mediated by oncogene-induced senescence (OIS), is thought to play a protective role in the development of PDAC. In the Kras-driven PDAC mouse model, Lesina et al. demonstrated that *RELA* reinforced OIS to inhibit carcinogenesis [36]. However, genetically disabling OIS can cause *RELA* to promote tumor proliferation; thus, revealing a dual role of *RELA* in PDAC carcinogenesis.

*NFKB1* and *IKBKG* are part of the NF-*κ*B signaling pathway. As a transcription factor, *NFKB1* is closely related to the risk of PDAC occurrence and prognosis [37]. Low expression of MUC4 inhibited the expression of *NFKB1*, thereby downregulating the NF-*κ*B signaling pathway to inhibit the migration and invasion of PDAC cells along the nerve [38]. The polymorphisms of *NFKB1* also significantly increase susceptibility to cancer in Asians [39], and several researchers have pointed out the important role of *NFKB1* as an inhibitor of PDAC [40]. *IKBKG* binds and regulates I*κ*B kinase (IKK), which inhibits NF-*κ*B activation and increases the cleavage of PARP and Caspase 3 in the apoptotic pathway to promote apoptosis in PDAC cells. It has also been reported that regulating the activity of *IKBKG* is used to promote the sensitivity of PDAC to gemcitabine [41]. The NF-*κ*B signaling pathway and TGF-*β* have a role in delaying the progression of pancreatic fibrosis [42], thereby inhibiting PDAC progression.

*JUN* may be involved in the growth of PDAC cells. It plays an important role in regulating the K-Ras and p38MAPKpathway by interfering with *JUN* and exerting anti-inflammatory activity and inhibiting PDAC metastasis [43]. *MAPK1* is an important regulatory factor in the MAPK signaling pathway, which greatly enhances the migration and invasion of PDAC cells for inducing EMT [44]. Therefore, inhibition of *MAPK1* expression is also a potential target for future oncological research. *AKT1* has been identified as an oncogene in a variety of cancers, including PDAC, which confirmed that activated *AKT1* accelerates the occurrence and development of PDAC and induces apoptosis of PDAC cells by inhibiting *AKT1* expression [45]. Phosphorylation of *AKT1* also increases the risk of cachexia in the PDAC population, which is strongly associated with disease prognosis [46].

*TP53* mutations occur in more than 75% of PC patients, and mutated *TP53* promotes EMT and tumor cell invasion [47]. *TP53* is a driver gene that is essential for the proliferation and metastasis of PDAC, and the expression of *TP53* results in shorter disease-free survival (HR: 1.33; 95% CI, 1.02-1.75; *P* = 0.04) [48]. In addition, some studies have found that the mutation of *TP53* is closely related to the occurrence of malignant intraductal papillary mucinous neoplasm (IPMN) [49]. Therefore, silencing or inactivation of *TP53* will prevent the further development of IPMN to PDAC and improve the prognosis of patients.

For the diagnostic value of the above genes in PDAC, we found that *RELA* had the highest value, which is consistent with previous findings. And the predictive value of the combined group was much higher than that of a single gene. However, this study failed to select more effective combined predictive markers because the predictive value of *AKT1* and *JUN* in the results is low, which may reduce the predictive value of the combined group, which is the direction we need to study in the future.

Similarly, in prognostic and survival analyses, we selected *RELA*, which has the highest diagnostic value, for prediction, and excitedly, it has a high value in predicting disease-specific survival and progress-free interval, even if it is not meaningful in overall survival. However, the derivation of the above predictive markers still needs to be further confirmed by experimental or clinical studies, which is also one of the limitations of this study.

### 4.3. Gene Ontology Interprets the Multifaceted Nature of USM

There are many transcription factors in the gene targets of USM for the treatment of PDAC, as well as in the binding processes of enzyme, transcription factor, and receptor protein. For example, myc-associated zinc-finger protein (MAZ) is the transcription factor involved in the transcription initiation and termination. Deregulation of MAZ expression is associated with the progression of PDAC and increases the CRAF-ERK signal. It is mediated through p21-activated protein kinase and protein kinase B (AKT) signaling cascades to enhance the invasion of PDAC cells [50].

USM inhibited the proliferation and induced apoptosis in human PC xenografts through various mechanisms, such as cell cycle arrest in the G2/M phase, downregulating the expression of phosphorylated Akt and mTOR, and regulating the PI3K/Akt/mTOR signaling pathway [7]. Previous studies have shown that KLTi reduces NF-*κ*B levels in the nucleus. Additionally, it reduces the expression of I*κ*B*α*, IKK, and EGFR in tumor cells and the overall cytoplasm. This corresponds to the role of KLTi at the nuclear and cytoplasmic levels [51]. Thus, the intervention of the binding of factors might have some interference effects on PDAC.

### 4.4. USM through Multiple Pathway Regulation for PDAC

Results from KEGG analysis showed that USM can act directly on PC, in addition to intervening in pathways that affect tumor development. This observation indirectly illustrates the important value of KLTi in the treatment of PDAC.

It has been proven that many malignant tumors are associated with virus infection. Studies have shown a correlation between hepatitis-B virus (HBV) infection and the occurrence of PC and poor prognosis. The X protein released by HBV significantly enhances cell proliferation and migration, induces EMT, upregulates PI3K-Akt and MAPK signaling pathways, renders PDAC malignant, and promotes disease progression [52].

Regulating the cell cycle also plays a role in the development of PDAC. A variety of genes and proteins are involved in this process. Usami et al. [53] observed that the class IIa HDACi could inhibit the activation of FOXO3, thus inhibiting the growth of PC cells. The combination of class IIa HDACi with the proteasome inhibitor carfilzomib could have a synergistic effect on the FOXO3 activation, thus, resulting in G1/S arrest in AsPC-1 cells.

Peripancreatic nerve invasion is an important oncological feature of PDAC and is closely related to disease prognosis. USM can also act on the neurotrophin signaling pathway to intervene in nerve invasion. Perineural invasion is associated with a variety of neurotrophic factors produced by neural tissue inside and outside the pancreas, which bind to specific receptors resulting in autophosphorylation and activation of multiple signaling pathways, such as MAPK PI3K-Akt and NF-*κ*B [54]. The nerve growth factor promotes the spread of PC cells by autocrine and/or paracrine mechanisms through MAPK-mediated phosphorylation [55]. It also activates the ERK/CD133 signaling cascade, resulting in enhanced tumor cell invasion, and plays a key role in the perineural invasion of PC [56]. Studies have confirmed that regulating the NF-*κ*B signaling pathway through activating IKK plays an important role in mediating EMT and inducing neural invasion [57].

The activation of the MAPK signaling pathway is crucial for PDAC proliferation and metastasis. This pathway is involved in the regulation of various biological activities through three major proteins, ERK1/2, p38MAPK, and MKK4 [58]. Yan et al. [59] compared the expression of p-ERK1/2 between cancerous pancreatic tissues and normal cells. They found that the expression of p-ERK1/2 in pancreatic tissues was significantly increased. In vivo and in vitro experiments confirmed that the inhibition of ERK1/2 expression reduced EMT, activated cancer-related autophagy, and decreased cell proliferation and migration in human PC cells. In another study [60], it was shown that the p38MAPK inhibitor, VCP979, could regulate the MAPK/NF-*κ*B signaling pathway, reduce inflammation, and inhibit EMT to exert an antitumor effect. Further, MKK4 was associated with the high proliferation of tumor cells and promoted the rapid proliferation of PDAC cells.

The PI3K-Akt signaling pathway is a key pathway that promotes tumor cell proliferation, invasion, metastasis, and drug resistance. As one of the substrates of Akt, Girdin enhanced phosphorylation of Akt and induced activation. Wang et al. [61] found that Girdin showed high expression in PDAC and was involved in the regulation of tumor cell metastasis, angiogenesis, and autophagy. Silencing of the Girdin gene resulted in decreased levels of p-Akt and p-PI3K and inhibition of the PI3K-Akt signaling pathway, thereby increasing apoptosis and inducing cell cycle arrest in tumor cells. PI3K-Akt signaling pathway is closely related to the abnormal expression of lncRNA. Studies [62] have shown that the expression of lncRNA small nucleolar RNA host gene1 elevates the expression of PI3K and phosphorylated Akt, which in turn activates the PI3K-Akt signaling pathway to promote cell proliferation, inhibits apoptosis, and enhances invasion in PDAC. The expression of lncRNA AB209630 inhibited the PI3K-Akt signaling pathway in gemcitabine-resistant PDAC cells and reduced the proliferation of resistant cells to improve the sensitivity to chemotherapy [63].

It is worth noting that both MAPK and PI3K-Akt are important signaling pathways for the transduction of membrane receptor signals into cells, and there exists an interaction of receptor signals in the two pathways [64]. Ras, an upstream molecule of MAPK, can induce the activation of Akt, and p38MAPK can act between PI3K and Akt and thus play an important role in Akt phosphorylation. Similarly, the activity of PI3K has an important induction effect on the activity of the Ras/MAPK pathway, and Akt can also negatively regulate the Ras/MAPK pathway by phosphorylating Raf [65]. PI3K-Akt and NF-*κ*B signaling pathways also have an interaction effect. Akt activates Ikk, by phosphorylation, then releases NF-*κ*B from the cytoplasm for nuclear translocation, activates downstream gene expression, and participates in the regulation of the NF-*κ*B pathway [66].

## 5. Conclusions

Through the network pharmacology, molecular docking, and database verification (GEO, TCGA, diagnostic ROC, and survival prognosis analysis), our study found that the USM in KLTi for PDAC could regulate the pancreatic cancer pathway and provide new diagnostic and predicted molecules for *RELA*, thus, providing scientific evidence for the rational application of KLTi for PDAC in clinical practice.

## Figures and Tables

**Figure 1:** Workflow of network pharmacology analysis.

**Figure 2:** Evaluation of pharmacological and toxicological parameters of main compounds from unsaponifiable matter (USM). ((a) Pharmacological and molecular properties of the main compounds in USM. (b) The toxicological parameters include hepatotoxicity, carcinogenicity, immunotoxicity, mutagenicity, cytotoxicity, and acute oral toxicity of the main compounds in USM. (c) The chemical structure and drug-likeness parameters of the main compounds extracted from USM. Red numbers represent drug-likeness values. MW: molecular weight; Hdon: hydrogen bond donor count; Hacc: hydrogen bond acceptor count; Rbon: rotatable bond count; LoaP: lipid-water partition coefficient).

**Figure 3:** Related targets in unsaponifiable matter (USM) and pancreatic ductal adenocarcinoma (PDAC). ((a) Compound-target network of USM. Blue hexagons represent targets; pink circles represent compounds. (b) Volcano plot of differentially expressed genes in PDAC. The abscissa represents the fold changes in gene expression, and the ordinate represents the statistical significance of the variations in gene expression. The red dots represent significantly differentially expressed genes. (c) Heat map of differentially expressed genes in PDAC).

**Figure 4:** The protein-protein interaction (PPI) network of unsaponifiable matter candidate genes against pancreatic ductal adenocarcinoma (PDAC). ((a) The interactive PPI network of unsaponifiable matter putative targets and PDAC-related targets. (b) PPI network of significant proteins extracted from (a). (c) PPI network of candidate unsaponifiable matter targets for PDAC therapy extracted from (b). DC: degree centrality; BC: betweenness centrality; CC: closeness centrality).

**Figure 5:** Unsaponifiable matter treatment of pancreatic ductal adenocarcinoma core protein-protein interaction network internal potential module network.

**Figure 6:** Gene ontology (GO) terms and KEGG pathway enrichment of candidate genes of unsaponifiable matter against pancreatic ductal adenocarcinoma. (The left side of the graph is the top GO name, the colors of the bars from orange to red represent the log10 (FDR) values (from small to large), and the longer bar represents the gene count of this GO. The size of the bubble represents the number of genes in the pathway, the colors from blue to red represent log10*P* values (from small to large), the vertical axis represents the top pathway name, and the horizontal axis represents the ratio of the overall input genes in the pathway).

**Figure 7:** Gene-pathway network of unsaponifiable matter against pancreatic ductal adenocarcinoma. (Yellow diamonds represent target genes, light blue squares represent pathways, and a bigger size represents a larger degree).

**Figure 8:** Molecular docking of compounds with targets.

**Figure 9:** RMSD plot during molecular dynamic simulations of compounds with targets.

**Figure 10:** Diagnostic ROC with targets. (The area value under the ROC curve is between 0.5 and 1. The closer the AUC is to 1, the better the diagnostic effect. Low accuracy of AUC between 0.5 and 0.7, certain accuracy of AUC between 0.7 and 0.9, and high accuracy of AUC above 0.9).

**Figure 11:** Survival and prognosis value of *RELA*.

**Table 1:** Description of potential module functions within protein-protein interaction network for unsaponifiable matter treatment of pancreatic ductal adenocarcinoma (top 3).

Color	GO	Description	Log10*P*
Red	GO:0003735	Structural constituent of ribosome	-29.7
	GO:0005198	Structural molecule activity	-21.6
	GO:0019843	rRNA binding	-11.2

Blue	GO:0019904	Protein domain-specific binding	-11.5
	GO:0043021	Ribonucleoprotein complex binding	-9.3
	GO:0031625	Ubiquitin protein ligase binding	-8.4

Green	GO:0031625	Ubiquitin protein ligase binding	-18.4
	GO:0044389	Ubiquitin-like protein ligase binding	-18.1
	GO:0019904	Protein domain-specific binding	-11.7

Purple	GO:0008134	Transcription factor binding	-13.8
	GO:0003682	Chromatin binding	-11.6
	GO:0001085	RNA polymerase II transcription factor binding	-9.8

Orange	GO:0003712	Transcription coregulator activity	-6.1
	GO:0031625	Ubiquitin protein ligase binding	-5.6
	GO:0044389	Ubiquitin-like protein ligase binding	-5.5

**Table 2:** Molecular docking results of compound-target.

Number	Compounds	Targets	Binding affinity (kcal/mol)
A	Stigmasterol	*JUN*	-9.4
B	Stigmasterol	*MAPK1*	-9.3
D	Stigmasterol	*RELA*	-7.61
C	Stigmasterol	*TP53*	-6.5
E	Isoarborinol	*JUN*	-7.4
F	Isoarborinol	*MAPK1*	-7.6
H	Isoarborinol	*RELA*	-7.25
G	Isoarborinol	*TP53*	-7.2

## Data Availability

All datasets presented in this study are available from the corresponding author upon request.
